This article has been retracted.

# Vitamin AD Drops are More Effective than Intramuscular Injection of Thymosin in Reducing the Rate of Growth Retardation in Children

**DOI:** 10.1155/2022/7799111

**Published:** 2022-08-11

**Authors:** Min Luo, Hui Zhang

**Affiliations:** ^1^Child Health Center, Shiyan Maternal and Child Health Hospital, Shiyan, Hubei, China; ^2^Department of Neonatology, Shiyan Maternal and Child Health Hospital, Shiyan, Hubei 442000, China

## Abstract

**Objective:**

To explore the effect of vitamin AD drops on growth retardation in children.

**Methods:**

From February 2020 to February 2021, 100 children with constipation and recurrent respiratory infections treated in our hospital were assigned to a vitamin AD drops group and intramuscular thymosin group, with 50 cases in each group. Outcome measures included mean height, body mass index (BMI), frequency of respiratory infections, increase in height and BMI, growth retardation, clinical effectiveness, immune function, medication compliance, and adverse responses.

**Results:**

The vitamin AD drops group showed higher mean height (*t* = 5.958, *P* < 0.05), greater body mass (*t* = 3.997, *P* < 0.05), and less frequency of respiratory infections than the intramuscular thymosin group (*t* = 26.564, *P* < 0.05). The vitamin AD drops group resulted in a lower ratio of height increase of >1 cm and a higher ratio of >2 cm as compared with the intramuscular thymosin group (*χ*^2^ = 8.167, *P* < 0.05). The vitamin AD drops group showed a lower ratio of weight gain of 0 and > 1 kg and a higher ratio of >2 kg versus the intramuscular thymosin group (*χ*^2^ = 4.058, *P* < 0.05). Vitamin AD drops resulted in a significantly lower growth retardation rate than intramuscular thymosin administration (*χ*^2^ = 5.530, *P* < 0.05). The vitamin AD drops group yielded markedly higher treatment efficiency in contrast to the intramuscular thymosin group (*Z* = 2.111, *P* < 0.05). The levels of CD3+CD4+, CD3+CD8+, CD4/CD8, IgA, IgG, and IgM in the two groups of patients after medication were higher than those before medication (*P* < 0.05), with higher levels in the vitamin AD drops group compared with the intramuscular thymosin group (*P* < 0.05). The vitamin AD drops group showed remarkably higher medication compliance in patients versus the intramuscular thymosin group (*Z* = 2.239, *P* < 0.05). The vitamin AD drops group experienced a significantly lower incidence of adverse reactions (*χ*^2^ = 4.396, *P* < 0.05).

**Conclusion:**

Vitamin AD drops are more effective than the intramuscular injection of thymosin in reducing the incidence of growth retardation in children.

## 1. Introduction

Short stature is defined as individuals of the same race, sex, and age whose height is less than 2 standard deviations from the mean height of the normal population, or less than the 3rd percentile (P3), in similar living environments. Currently, growth hormone therapy is effective in treating short stature, but it is costly and associated with side effects. In children under P3 height, excluding those with growth hormone deficiency and idiopathic dwarfism due to the effects of related diseases, growth hormone therapy is mostly used [1, 2].

Furthermore, diseases such as repeated respiratory tract infections and constrictions are far more common in infants and children, and nutrients such as zinc and vitamin D in infants and children are easily deficient under various factors during the growth course, leading to various diseases and jeopardizing their development [3].

Children with height between the 3rd and 10th percentile (P3 to P10) have short stature and growth retardation but fail to reach the diagnostic criteria for dwarfism and growth hormone therapy is discouraged, for which modern medicine only provides nutrition and exercise guidance, but the results are unfavorable. These children exhibit thinness, yellowish complexion, poor appetite, partial and picky eating, loose stools, thick and greasy tongue coating, inactivity, and poor sleep, which are consistent with spleen deficiency with dampness in the traditional Chinese medicine (TCM) theory [4]. Research has revealed that children with short stature are commonly deficient in 25 hydroxyvitamins and trace elements of zinc compared to normal children of the same age [5]. Therefore, early diagnosis of bone mineral density deficiency in children with growth retardation is merited for effective clinical treatment. Bone mineral density values provide an accurate evaluation of the mineral content of the bones and facilitate the understanding of the skeletal development of the child, which plays a crucial role in bone density testing. Vitamin A is a micronutrient and vitamin D provides the body with the required nutrients and plays a role in the regulation of calcium metabolism [6]. Clinical research has demonstrated significantly lower vitamin D levels in children with growth retardation compared to normal children, but related current clinical reports are scarce [7].

Vitamin AD drops are a compound preparation for vitamin A and vitamin D supplementation, they regulate the immune system, and enhance the anti-infection ability of the body [8]. Tiaozhong Zhuyun decoction strengthens the spleen and benefits the qi. This study statistically analyzed the clinical data of 100 children with constriction in our hospital from February 2020 to February 2021 and explored the effect of vitamin AD drops on growth retardation in children.

## 2. Materials and Methods

### 2.1. General Information

From February 2020 to February 2021, 100 children with constipation and recurrent respiratory infections treated in our hospital were assigned to a vitamin AD drops group and an intramuscular thymosin group, with 50 cases in each group. The randomization was carried out using an online web-based randomization tool (https://www.randomizer.org/). For concealment of allocation, the randomization procedure and assignment were managed by an independent research assistant who was not involved in screening or evaluation of the participants.

In the vitamin AD drops group, there were 21 females and 29 males, aged 1–14 (7.02 ± 1.32) years, 24 cases with a disease duration of 1–2 years, and 26 cases with 3–4 years; there were 44 cases of repeated upper respiratory tract infections, 41 cases of anorexia, and 9 cases of malnutrition. In the intramuscular thymosin group, there were 20 females and 30 males, aged 1–14 (7.10 ± 1.52) years, 23 cases with a disease duration of 1–2 years, and 27 cases with 3–4 years; there were 43 cases of repeated upper respiratory tract infections, 40 cases of anorexia, and 11 cases of malnutrition. The patient characteristics between the two groups were comparable (*P* > 0.05).

The original sample size calculation estimated that 50 patients in each group would be needed to detect a 3-point difference between the groups in a 2-sided significance test with a power of 0.8 and an alpha error level of 0.05. Undersigned informed consent was obtained from patients prior to enrollment in this study. The study protocol was approved by the hospital's ethics committee, ethics number: SU-EU20200204. All the processes were in accordance with the Declaration of Helsinki's ethical guidelines for clinical research.

#### 2.1.1. Inclusion Criteria

(1) All had complete medical records; (2) children with birth length ≥50 cm, body mass ≥2.5 kg, normal intelligence, and no congenital organic disease; (3) children with height growth curves between P3 and P10; (4) children with growth retardation: 5 cm < 6 cm/year growth rate; (5) bone age lagged behind the actual age (≤1 year); (6) children with chronic anorexia, picky eating, or low food intake; (7) patients who provided informed consent and cooperated with treatment.

#### 2.1.2. Exclusion Criteria

(1) Patients with acute myocardial infarction; (2) patients with arrhythmia; (3) patients with cardiopulmonary insufficiency. (4) patients with thyroid dysfunction, skeletal disorders, genetic metabolic diseases, Turner syndrome, precocious puberty, early menarche, early breast development, pituitary tumors, and other organic pathologies that cause growth retardation; (5) patients with treatment adherence.

### 2.2. Method

#### 2.2.1. Intramuscular Injection of Thymosin Group

The children were intramuscularly administered with 1 mg of thymosin, twice a week. With 1 month as one treatment cycle, the duration was 3 courses.

#### 2.2.2. Vitamin AD Drops Group

The children were given one pill of vitamin AD drops once on alternate days. With 1 month as one treatment cycle, the duration was 3 courses.

The two groups received Tiaozhong Zhuyun granules. The ingredients of the granules include 12 g of Pseudostellariae Radix, 8 g of Poria, 9 g of Atractylodis Macrocephalae Rhizoma and Atractylodis Rhizoma, 10 g of Dioscoreae Rhizoma, 6 g of *Pinellia tuberifera*, 9 g of tangerine peel, 8 g of fried white lentils, Coicis Semen and Galli gigeriae endothelium corneum, 6 g of Amomi Fructus, 3 g of licorice, and 2 g of *Stevia rebaudiana*. The granules were administered with one dose daily for 5 days a week. With 3 months as one treatment cycle, the duration was 2 courses.

### 2.3. Observation Indicators

The patients were followed up for 3 months. (1) Mean height, body mass index, and frequency of respiratory infections; (2) height and weight gain; (3) growth retardation; (4) immune function, including CD3+CD4+, CD3+CD8+, CD4/CD8, and other T cell subsets, and IgA, IgG, IgM, and other serum immunoglobulin indicators; before and after treatment, 9 mL of morning fasting venous blood was collected from patients and centrifuged to obtain the serum, which was stored at −20°C for assays. The rate method was adopted for measurement using a Beckman fully automated biochemistry analyzer (Beckman Kulk, USA); (5) medication compliance; (6) adverse reactions.

### 2.4. Efficacy Evaluation Criteria

Markedly effective: the clinical manifestations and respiratory infections after medication have been significantly reduced, with the frequency of less than 0.66 times one month, and no recurrence was observed within 3 months; effective: the clinical manifestations and respiratory infections after medication have been significantly reduced, with the frequency of 0.66∼2.65 times/month, and no recurrence was observed within 3 months; ineffective: the clinical manifestations and respiratory tract infections worsened after the medication, with a frequency of 2.65 times one month, and recurrence was observed within months [9].

### 2.5. Statistical Analysis

All the data analyses were performed by SPSS21.0. The count data were expressed as rates and analyzed using the *χ*^2^ test or rank sum test. Measurement data were expressed as $\bar{x}\pm s$ and examined using the *t*-test or *F* test. *α* = 0.05 was assumed to be significant.

## 3. Results

### 3.1. Comparison of Mean Height, BMI, and the Frequency of Respiratory Infections

The vitamin AD drops group showed higher mean height (*t* = 5.958, *P* < 0.05), greater body mass (*t* = 3.997, *P* < 0.05), and less frequency of respiratory infections than the intramuscular thymosin group (*t* = 26.564, *P* < 0.05). (Table1).

### 3.2. Comparison of Growth in Height, BMI, and Growth Retardation

The ratio of height increase >1 cm was lower in the vitamin AD drops group and higher in the intramuscular thymosin group (2 = 8.167, *P* < 0.05); the ratio of weight gain of 0 and > 1 kg was lower in the vitamin AD drops group and higher in the intramuscular thymosin group (2 = 4.058, *P* < 0.05), and the growth retardation rate was lower in the vitamin AD drops group (2 = 5.530, *P* < 0.05). (Table 2).

### 3.3. Comparison of Clinical Efficacy

The vitamin AD drops group yielded markedly higher treatment efficiency in contrast to the intramuscular thymosin group (*Z* = 2.111, *P* < 0.05) (94.00% (47/50) vs 80.00% (40/50)) (*Z* = 2.111, *P* < 0.05). (Table 3).

### 3.4. Comparison of Immune Function

The levels of CD3+CD4+, CD3+CD8+, CD4/CD8, IgA, IgG, and IgM in the two groups of patients after medication were higher than those before medication (*P* < 0.05), with higher levels in the vitamin AD drops group compared with the intramuscular thymosin group (*P* < 0.05, Tables 4 and 5).

### 3.5. Comparison of Medication Compliance

The vitamin AD drops group showed remarkably higher medication compliance in patients versus the intramuscular thymosin group (90.00% (45/50) vs 66.00% (33/50)) (*Z* = 2.239, *P* < 0.05) (Table 6).

### 3.6. Comparison of Adverse Reactions

The vitamin AD drops group experienced a significantly lower incidence of adverse reactions (2.00% (1/50) vs 16.00% (8/50)) (*χ*^2^ = 4.396, *P* < 0.05). (Table 7).

## 4. Discussion

Since the publication of the guidelines for the diagnosis and treatment of children with short stature by the Chinese Academy of Pediatrics, children with short stature below the 3rd percentile (P3) in height have received widespread attention, and 60%–80% of these children with growth retardation are classified as idiopathic short stature (ISS) whose pathogenesis remains poorly understood [10]. Infants and young children are extremely susceptible to various factors that lead to insufficient intake of nutrients [11]. The current consensus is to use growth hormones for disease management. However, due to the high price of growth hormone preparations, the need for long-term injections, and unknown side effects, the widespread use of the growth hormone is largely limited. Modern medical nutrition and exercise guidance for short stature is insufficient, and some cases are characterized by lagging growth, bloating, partiality, and picky eating [12]. Vitamin AD drops contain vitamin A and vitamin D, among which vitamin D promotes the body's absorption of calcium and facilitates the growth and development of children [1]. Studies have shown [13, 14] that vitamin AD drops play a positive role in the prevention of upper respiratory tract infections and provide favorable conditions for the growth and development of children.

In TCM, “short stature” is included in the category of “five growth delays.” The present study revealed that spleen deficiency is common in children with growth retardation according to clinical practice. Children require high nutritional needs during growth and development, and adequate nutritional supply necessitates a strong spleen and stomach to properly transport and absorb water and grain essences; thus, tonifying the spleen and stomach is the key to treatment. In this formula, Pseudostellariae Radix and Atractylodis Macrocephalae Rhizoma strengthen the spleen and tonify qi, while Atractylodis Rhizoma, Dioscoreae Rhizoma, tangerine peel, Poria, Dioscoreae Rhizoma, white lentils, and Coicis Semen invigorate the spleen and remove dampness. Amomi Fructus and Galli gigeriae endothelium corneum stimulate the spleen and help digestion, and licorice tonifies the middle, strengthens the qi, and harmonizes the medicines. Modern pharmacological studies have shown that Liujunzi decoction promoted the absorption and secretion function of the small intestine and the secretion function of the stomach and pancreas. Pseudostellariae Radix is immune-promoting and rich in zinc, and Atractylodis Macrocephalae Rhizoma and Atractylodis Rhizoma are both rich in vitamin A. Vitamin A contributes to the better functioning of vitamin D. The whole formula is balanced and has the effect of strengthening the spleen, benefiting Qi to help growth, and harmonizing the stomach to help transportation of qi and promote absorption [15].

Vitamin AD drops resulted in a significantly lower growth retardation rate than intramuscular thymosin administration (*χ*^2^ = 5.530, *P* < 0.05). The vitamin AD drops group yielded markedly higher treatment efficiency in contrast to the intramuscular thymosin group (*Z* = 2.111, *P* < 0.05). The levels of CD3+CD4+, CD3+CD8+, CD4/CD8, IgA, IgG, and IgM in the two groups of patients after medication were higher than those before medication (*P* < 0.05), with higher levels in the vitamin AD drops group compared with those in the intramuscular thymosin group (*P* < 0.05). The vitamin AD drops group showed remarkably higher medication compliance in patients versus the intramuscular thymosin group (*Z* = 2.239, *P* < 0.05). The vitamin AD drops group experienced a significantly lower incidence of adverse reactions (*χ*^2^ = 4.396, *P* < 0.05). The results of the present study showed that the vitamin AD drops group showed higher mean height (*t* = 5.958, *P* < 0.05), greater body mass, and less frequency of respiratory infections than the intramuscular thymosin group. Moreover, the vitamin AD drops group resulted in a lower ratio of height increase>1 cm and a lower ratio of weight gain 0 and > 1 kg, and a higher ratio of>2 cm and a ratio of >2 kg as compared with the intramuscular thymosin group. Moreover, the vitamin AD drops group yielded markedly higher total treatment efficiency in contrast to the intramuscular thymosin group (94.00% (47/50) vs 80.00% (40/50)). All the abovementioned results were in line with the previous studies [16, 17], which may be attributed to the key role of vitamins A and D. Vitamin A ensures embryonic development, and bone reproduction and growth, presents in both osteoblasts and osteoclasts, inhibits osteoclast activity, activates osteoclasts, and facilitates skeletal growth, development, and bone formation [18]. Vitamin D regulates bone metabolism, maintains normal cellular activity, and increases calcium absorption, thereby facilitating bone development and growth [19]. Vitamin A affects thyroid and the growth hormone-insulin growth factor axis function, which consequently regulates bone metabolic indexes [20], and vitamin D regulates calcium and phosphorus metabolism, facilitates the promotion of calcium and phosphorus absorption, provides essential minerals for normal bone tissue, and contributes to osteocalcin and osteoclast synthesis [21, 22].

Previous studies reported [23–26] that vitamin D effectively regulated the human immune function. The present study showed that after medication, the levels of CD3+CD4+, CD3+CD8+, CD4/CD8, IgA, IgG, and IgM in the two groups of patients after medication were higher than those before medication, with a higher level in the vitamin AD drops group compared with the intramuscular thymosin group, and the vitamin AD drops group showed higher medication compliance than the intramuscular thymosin group (90.00% (45/50) vs 66.00% (33/50)); the vitamin AD drops group experienced a considerably lower adverse reaction rate (2.00% (1/50) vs 16.00% (8/50)), which were consistent with the results of the prior study [27]. It is presumably attributed that vitamin D in AD drops enhances the immune function of the monocyte-macrophage system, activates T cells, provides favorable conditions for monocytes-macrophages, and induces the production of the tumor necrosis factor and interleukin [28–30]. Thymosin is a biologically active peptide extracted from calf thymus tissue that regulates the immune system and boosts body disease resistance but fails to provide sufficient vitamin A required by the body, resulting in a somber effect compared with vitamin AD drops [31, 32].

This trial was a guideline for the treatment of vitamin AD in patients with growth retardation. However, the present study may compromise the quality of the results due to the small number of samples included. Therefore, more samples should be included in future studies for an in-depth study to improve the accuracy of the results. In the future, a greater sample size and longer follow-up studies will be necessary to give more authentic evidence for clinical practice. Collectively, vitamin AD drops may provide a viable treatment alternative for growth retardation.

## Figures and Tables

**Table 1:** Comparison of average height, BMI, and frequency of respiratory infections ($\bar{x}\pm s$).

Groups	*n*	Average height (cm)	BMI (kg)	Frequency of respiratory infections (time/month)
Vitamin AD drops group	50	118.84 ± 9.67	26.84 ± 5.95	0.64 ± 0.12
Intramuscular thymosin group	50	108.20 ± 8.12	22.62 ± 4.51	2.03 ± 0.35
*t*		5.958	3.997	26.564
*P*		<0.001	<0.001	<0.001

**Table 2:** Comparison of growth in height, BMI, and growth retardation (*n* (%)).

Groups	*n*	Growth in height		Growth in BMI			Growth retardation
Vitamin AD drops group		>1 cm	>2 cm	0	>1 kg	>2 kg	
Intramuscular thymosin group	50	13 (26.00)	37 (74.00)	0 (0)	17 (34.00)	33 (66.00)	0 (0)
Groups	50	27 (54.00)	23 (46.00)	1 (2.00)	26 (52.00)	23 (46.00)	7 (14.00)
*χ* ^2^		8.167		4.058			5.530
*P*		0.004		0.044			0.019

**Table 3:** Comparison of clinical efficacy (*n* (%)).

Groups	*n*	Markedly effective	Effective	Ineffective	Total effectiveness
Vitamin AD drops group	50	24 (48.00)	23 (46.00)	3 (6.00)	47 (94.00)
Intramuscular thymosin group	50	16 (32.00)	24 (48.00)	10 (20.00)	40 (80.00)
*Z*					2.111
*P*					0.035

**Table 4:** Comparison of immune function ((%), $\bar{x}\pm s$).

Groups	*n*	Time	CD_3_^+^CD_4_^+^	CD_3_^+^CD_8_^+^	CD_4_/CD_8_
Vitamin AD drops group	50	Before medication	22.02 ± 4.14	33.42 ± 5.24	1.02 ± 0.26
		After indication	26.23 ± 5.24	38.75 ± 4.41	1.52 ± 0.41

Intramuscular thymosin group	50	Before medication	21.75 ± 4.06	33.75 ± 5.03	1.03 ± 0.30
		After indication	23.45 ± 4.15	34.45 ± 4.65	1.12 ± 0.30

**Table 5:** Comparison of the immune function (g/L, $\bar{x}\pm s$).

Groups	*n*	Time	IgA	IgG	IgM
Vitamin AD drops group	50	Before medication	1.02 ± 0.30	7.25 ± 1.06	1.02 ± 0.35
		After indication	1.52 ± 0.25	8.32 ± 1.14	1.35 ± 0.28

Intramuscular thymosin group	50	Before medication	1.03 ± 0.30	7.15 ± 1.25	1.05 ± 0.28
		After indication	1.10 ± 0.30	7.42 ± 1.48	1.12 ± 0.31

**Table 6:** Comparison of medication compliance (*n* (%)).

Groups	*n*	Totally compliant	Partially compliant	Completely incompliant	Total compliance
Vitamin AD drops group	50	22 (44.00)	23 (46.00)	5 (10.00)	45 (90.00)
Intramuscular thymosin group	50	16 (32.00)	17 (34.00)	17 (34.00)	33 (66.00)
*Z*					2.239
*P*					0.025

**Table 7:** Comparison of adverse reactions (*n* (%)).

Groups	*n*	Nausea and vomiting	Itchy skin	Constipation	Dry mouth	Headache	Total incidence
Vitamin AD drops group	50	1 (2.00)	0 (0)	0 (0)	0 (0)	0 (0)	1 (2.00)
Intramuscular thymosin group	50	3 (6.00)	1 (2.00)	2 (4.00)	1 (2.00)	1 (2.00)	8 (16.00)
*χ* ^2^							4.396
*P*							0.036

## Data Availability

All data generated or analyzed during this study are included in this published article.
